RETRACTED

# *miRNA-148b* regulates radioresistance in non-small lung cancer cells via regulation of MutL homologue 1

**DOI:** 10.1042/BSR20150300

**Published:** 2016-06-30

**Authors:** Guangsheng Zhai, Gaozhong Li, Bo Xu, Tongfu Jia, Yinping Sun, Jianbo Zheng, Jianbin Li

**Affiliations:** * Department of Radiotherapy, The Tumor Hospital of Shandong Province, No. 440 of Jiyan Road, Ji'nan 250000, Shandong Province, China; † Department of Radiotherapy, The Central Hospital of Zibo, No. 54 of Gongqingtuan West Road 54, Zhangdian District, Zibo 255000, Shandong Province, China; ‡ Division of Gastroenterology, Department of Medicine, The Second Hospital of Shandong University, No. 54 of Gongqingtuan West Road 54, Zhangdian District, Zibo 255000, Shandong Province, China; § No. 1 Oncology Department, The Central Hospital of Zibo, No. 54 of Gongqingtuan West Road 54, Zhangdian District, Zibo 255000, Shandong Province, China; ║ No. 3 Oncology Department, The Central Hospital of Zibo, No. 54 of Gongqingtuan West Road 54, Zhangdian District, Zibo 255000, Shandong Province, China; ¶ Department of Urology Surgery, The Central Hospital of Zibo, No. 54 of Gongqingtuan West Road 54, Zhangdian District, Zibo 255000, Shandong Province, China

**Keywords:** lung cancer, *miR-148b*, MutL homologue 1 (MLH1), radioresistance

## Abstract

Radioresistance represents a major obstacle in cancer treatment, the underlying mechanism of which is complex and not well understood. *miR-148b* has been reported to be implicated regulating radioresistance in lymphoma cells. However, this function has not been investigated in lung cancer cells. Microarray analysis was performed in A549 cells 48 h after exposure to 8 Gy of γ-irradiation or sham irradiation to identify differentially expressed miRNAs. *miR-148b* mimic and inhibitor were transfected, followed by clonogenic survival assay to examine response to irradiation in A549 cells. Western Blot and luciferase assay were performed to investigate the direct target of *miR-148b*. Xenograft mouse models were used to examine *in vivo* function of *miR-148b*. Our data showed that expression of *miR-148b* was significantly down-regulated in both serum and cancerous tissues of radioresistant lung cancer patients compared with radiosensitive patients. Overexpression of *miR-148b* reversed radioresistance in A549 cells. MutL homologue 1 (MLH1) is the direct target of *miR-148b* which is required for the regulatory role of *miR-148b* in radioresistance. *miR-148b* mimic sensitized A549 xenografts to irradiation *in vivo*. Our study demonstrated that *miR-148b* regulates radioresistance of lung cancer cells by modulating MLH1 expression level. *miR-148b* may represent a new therapeutic target for the intervention of lung cancer.

RETRACTED

## Abstract (precis)

*miR-148b* regulates radioresistance of lung cancer cells by modulating MLH1 expression level.

## INTRODUCTION

Lung cancer is one of the leading causes of cancer-related deaths worldwide [1]. Non-small cell lung cancer (NSCLC) represents the most common type of lung cancer and accounts for approximately 80% of all lung cancer cases [2,3]. The 5-year overall survival rate of NSCLC cases is lower than 15% [3,4]. Approximately 40% of NSCLC patients have unresectable stage III disease or medically inoperable disease [5].

Radiotherapy has been regarded as one of the main treatment strategies for NSCLC. However, a large proportion of NSCLC patients are resistant to radiotherapy, which significantly limits its therapeutic effects and induces the local recurrence of NSCLC [6,7]. Although, it is generally thought to be due to tumour heterogeneity related to cell of origins, pathology, aetiology and molecular/genetic pathogenesis [8], the underlying mechanism remains unclear. Therefore, there is an urgent need to develop novel approaches for the intervention of NSCLC, such as targeted gene treatment as a radiosensitizer.

miRNAs is an abundant class of conservative and small non-coding RNAs which post-transcriptionally regulate gene by targeting mRNA for degradation or inhibition of translation [9]. miRNAs are implicated in regulating diverse tumorigenic processes, such as in cell apoptosis, cell proliferation, stress response and metabolism, etc., and have been found to be dysregulated in a wide variety of cancer types, including lung cancer [10–12]. Previous studies have shown that some miRNAs may be involved in modulating the sensitivity of cancer cells to radiotherapy and dysregulation of miRNA function might contribute to the acquisition of radioresistance, particularly in lung cancer [13–15].

Aberrant expression of *miR-148b* has been found in many cancer types, including breast cancer, prostate cancer, lung cancer, etc. [16–18]. In particular, *miR-148b* has been reported to be down-regulated in NSCLC and associated with poor survival [19] and it may function as a tumour suppressor in NSCLC by targeting carcinoembryonic antigen (CEA) [18]. Recently, it has been shown that *miR-148b* can reverse cisplatin-resistance in NSCLC via down-regulating DNA (cytosine-5)-methyltransferase 1 (DNMT1) expression [20]. Up-regulation of *miR-148b* has been observed in human endothelial cells after ionized radiation [21].

In the present study, we investigated the potential role of *miR-148b* in regulating radioresistance in NSCLC, the underlying mechanism and the potential clinical values using xenograft mouse models.

RETRACTED

## MATERIALS AND METHODS

### Cell culture and treatment

Human lung cancer cell line A549 (A.T.C.C.) was cultured in basal medium supplemented with 10% serum at 37°C and 5% CO_2_. These cells were tested mycoplasma free.

### Human samples

All the cancer samples and normal tissues were retrieved from The Tumor Hospital of Shandong Province. All tissues were immediately snap-frozen in liquid nitrogen and stored at −80°C until use. In addition, the patients with any other tumour were excluded from the study. Serum samples were extracted from whole blood after centrifugation (2800 ***g***, 10 min) and stored at −80°C until further processing. The present study was approved by The Tumor Hospital of Shandong Province and written informed consent was obtained from all patients.

### miRNA sequencing

A549 cells were seeded in six-well plates and exposed to 8 Gy of **γ**-irradiation or sham irradiation. After 48 h, these samples were lysed using Trizol reagent for total RNA collection. Subsequently, miRNA sequencing was performed using the Illumina sequencing platform single-end sequencing mode to conduct high-throughput sequencing for the four samples (Genenergy); each sample had three parallel groups. Differences between the groups were determined using the DESeq statistical tests of R software (genetic screening criteria: *P* ≤ 0.05 and fold difference in expression ≥ 1.5). Differential expression of miRNA between irradiated and nonirradiated cells was analysed after the sequencing was proofread using the genome and miRBase databases.

### Plasmids and cell transfection

Cells in exponential growth phase were prepared for cell transfection. Transfection of *miR-148b* inhibitor, *miR-148b* mimic and its non-specific control (Invitrogen) were performed according to the manual provided with the siPORTM NeoFXTM Transfection Agent (Ambion). pLenti-C-Myc-DDK MLH1 cDNA (RC201607L1) and shRNA plasmid (TL320419) targeting MutL homologue 1 (MLH1) were obtained from Origene. cDNA transfections were performed with Lipofectamine LTX reagent (Invitrogen) as per manufacturer's protocol.

### Viral transductions and stable selections

For lentivirus production, 1 μg of pLenti-C-Myc-DDK cDNA or shMLH1 plasmid together with 1 μg of helper plasmids (0.4 μg of pMD2G and 0.6 μg of psPAX2) were transfected into 293FT cells (A.T.C.C.) with Effectene reagent (Qiagen). Viral supernatants were collected 48 h after transfections and cleared through a 0.45 μm filter. Cells were infected with viral supernatants containing 4 μg/ml Polybrene (Sigma–Aldrich) and selected with puromycin for 7 days.

### Real-time PCR

The cells or spheroids were harvested after the transfection and the RNA was isolated using TRI reagent (Sigma–Aldrich). Ten nanograms of RNA were used for reverse transcription using the TaqMan MicroRNA RT Kit (Applied Biosystems, Life Technologies). Briefly, 5 μl of the RNA was added to 10 μl of the master mix containing 0.15 μl of dNTP (100 nM), 1 μl of multiscribe enzyme (50 units/μl), 1.5 μl of 10× RT-puffer, 0.19 μl of RNAse inhibitor (20 units/μl), 4.16 μl of RNAse free H_2_O and 3 μl of primers (*miR-200a/b/c*, *miR-141*). The conditions for the reverse transcription were 30 min at 16°C, 30 min at 42°C and 5 min at 85°C. Quantitative real-time PCR of the individual miRNAs was performed in a total volume of 10 μl containing 5 μl of TaqMan master mix, 3.17 μl of RNAse free H_2_O, 0.5 μl of TaqMan primer and 1.33 μl of cDNA. The PCR was performed in quadruple in a Rotor-Gene Corbett 6000 Q PCR (Life Science). The conditions for the reaction were: 2 min at 50°C, 10 min at 95°C, cycling (50 repeats): step 1–15 s at 95°C, step 2–60 s at 60°C. The data were collected and analysed using the quantitative Rotor-Gene software. The miRNA levels were normalized to the stable internal control miRNA RNU 6B using the algorithm of Pfaffl.

RETRACTED

### Colony formation assay

Cells were trypsinized and seeded in six-well plates at density of 1000 cells/well in triplicates immediately after exposure to γ-radiation. The cells were incubated for 1 week and then washed with PBS for three times, fixed with 4% paraformaldehyde for 15 min, and stained with 0.1% crystal violet (Sigma–Aldrich) solution for 30 min. After these, the colonies were carefully washed with PBS until the background is clear. Colony formation efficiency was calculated as colony number divided by 1000 and normalized to scramble or control vector cells.

### Immunoblot analysis

Total cell lysates were prepared by harvesting cells in Laemmli SDS reducing buffer [50 mM Tris/HCl (pH 6.8), 2% SDS and 10% glycerol], boiled and resolved on an 8–10% polyacrylamide gel, and transferred to polyvinylidinefluoride. Antibodies against MLH1 (Abcam) and β-actin (Sigma–Aldrich) were used. The blots were incubated with horseradish-peroxidase-conjugated donkey anti-rabbit or anti-mouse IgG (Santa Cruz Biotechnology) at a dilution of 1:5000 and detected with SuperSignal West Pico or Femto Chemiluminescent Substrate Kit (Thermo Scientific).

### γ-H2AX assay

Cells were exposed to 2 Gy of γ-radiation and were fixed using 3.7% paraformaldehyde for 10 min, permeabilized with 0.5% Triton X-100 in PBS on ice for 5 min and incubated with blocking solution (10% goat serum and 3% BSA in PBS containing 0.1% Triton X-100) for 30 min. Cells were then incubated with primary antibodies diluted in blocking solution for an hour. Anti-γ-H2AX antibody (1:100, Abcam, ab18311) was used. After incubation with secondary antibodies labelled with Alexa Fluor-568 (1:400, Invitrogen), slides were mounted with ProLong Gold Antifade Reagent with DAPI (Life Technologies). Cells were observed under a fluorescence microscope, Axiovert 200 M (Carl Zeiss). To quantify the number of γ-H2AX foci, at least 100 nuclei were analysed from each sample.

RETRACTED

### Luciferase assay

Two hundred and fifty nanograms of pGL3 reporter vector carrying the WT or mutant *miR-148b*-binding site (see plasmid construct, Figure 3A), 25 ng of the phRL-SV40 control vector (Promega) and 100 nM miRNA precursors or scrambled sequence miRNA control (Ambion) were co-transfected into HEK293 cells in 24-well plates. Firefly luciferase activity was measured with a Dual Luciferase Assay Kit (Promega) 24 h after transfection and normalized with a Renilla luciferase reference plasmid.

### Immunohistochemistry staining

The paraffin-embedded sections were subjected to antigen retrieval by heating the slides in a microwave at 100°C for 10 min in 0.1 M citric acid buffer (pH 6.0), and then incubated with corresponding antibodies at 4°C overnight. After secondary antibody incubation at room temperature for 1 h, the slides were developed in 0.05% diaminobenzidine containing 0.01% hydrogen peroxidase.

### Xenograft experiments

All animal experiments were approved by Institutional Animal Care and Use Committee of National Cancer Center. Control or *miR-148b* mimic transfected A549 cells (2×10^6^ cells/injection) were subcutaneously injected into both flanks of 5 weeks old female nude mice group. Tumour volumes were measured 3 weeks after exposure to 8 Gy of γ-radiation using calliper and determined by a formula [volume=(length × width^2^)/2] from day 3 to day 21 post implantation. The results were expressed as mean tumour volumes with S.D.

### Statistical analysis

Quantitative data are expressed as mean ± S.D. Statistical significance was assessed by the Student's *t* test. Differences were considered to be significant when *P*<0.05.

## RESULTS

### *miR-148b* expression is negatively related to radioresistance in lung cancer

In order to identify the miRNAs implicated in lung cancer radiosensitivity, miRNA sequencing was used to monitor their expression in A549 cells 48 h after radiation treatment. A549 has been demonstrated to be a radioresistant cell line before [22]. The results showed that radiation affected the expression of various miRNAs in A549 cells. Supplementary Figure S1(A) lists the top nine miRNAs that showed considerable up-regulation/down-regulation after irradiation. *miR-148b* was selected as the target miRNA as it showed greatest fold change in expression before and after irradiation. In addition, the difference in this expression was statistically significant before and after irradiation in A549 cells (*P*=0.0003) as confirmed by quantitative real-time PCR (Supplementary Figure S1B). *miR-148b* expression was analysed in lung cancerous tissues and matched non-cancerous tissues as well as serum from 20 CRC patients. The results showed lower expression of *miR-148b* in tumour tissues than in normal tissues (Figures 1A and 1C). Additionally, *miR-25* expression was also related to radiotherapy sensitivity. As shown in Figures 1(B) and 1(D), its expression was significantly lower in both tumour and serum samples of radioresistant patients than in radiosensitive counterparts. Therefore, dysregulation of *miR-148b* expression may be associated with radioresistance in lung cancer.

RETRACTED

**Figure 1:** *miR-148b* expression is negatively related to radioresistance in lung cancer (**A** and **C**) Quantitative real-time PCR analysis of relative *miR-148b* expression in serum (A) and tissue (C) of lung cancer patients (*n*=20) and healthy controls (*n*=20). (**B** and **D**) Quantitative real-time PCR analysis of relative *miR-148b* expression in serum (B) and tissue (D) of radiosensitive patients (*n*=15) and radioresistant patients (*n*=15). (A–D) Data represent mean ± S.D. ****, *P*<0.0001.

### *miR-148b* modulates radiosensitivity in lung cancer cells

To investigate whether *miR-148b* is involved in regulating radiosensitivity in lung cancer cells, we transfected *miR-148b* mimic or inhibitor into A549 cells which led to a significant increase or decrease in *miR-148b* expression (Figure 2A). Clonogenic survival assay showed that effective up-regulation or down-regulation of *miR-148b* significantly inhibited or promoted cell survival in A549 cells compared with control cells after exposure to 4 Gy of γ-radiation. To further elucidate the regulatory role of *miR-148b* in radioresistance, DNA double-strand breaks (DSBs) were measured and quantified using γ-H2AX foci staining. Compared with control cells, significantly more γ-H2AX foci persisted 6 h after irradiation in cells transfected with *miR-148b* mimic. On the contrary, significantly fewer foci persisted 2 and 6 h after irradiation in cells transfected with *miR-148b* inhibitor (Figure 2C). This suggests that *miR-148b* regulates radioresistance through mediating DNA damage repair (DDR).

**Figure 2:** *miR-148b* modulates radiosensitivity in lung cancer cells (**A**) Quantitative real-time PCR analysis of relative *miR-148b* expression in A549 cells transfected with *miR-148b* mimic or *miR-148b* inhibitor. Data represent mean ± S.D., *n*=3. **, *P*<0.01. (**B**) Clonogenic survival in control, mimic or inhibitor transfected cells after exposure to 4 Gy of γ-radiation. Survival was normalized to unirradiated control cells. Data represent mean ± S.D., *n*=3. **, *P*<0.01; ***, *P*<0.001. (**C**). DNA damage was assessed by γ-H2AX foci staining. A549 cells transfected with *miR-148b* mimic or inhibitor were irradiated with 2 Gy of γ-radiation, stained with γ-H2AX antibody at subsequent time intervals, and γ-H2AX foci were counted. *, *P*<0.05 compared with control transfected cells. To quantify the number of γ-H2AX foci, at least 100 nuclei were analysed from each sample.

RETRACTED

### *miR-148b* directly targets the 3’-UTR of MLH1 and regulates its expression level in lung cancer cells

To explore potential gene targets of *miR-148b* that may be involved in this effect, we examined for putative targets using miRNA target prediction programmes and MLH1 showed up as one of the hits that are most prevalent and this protein has been reported to play a role in regulating radioresistance in colon cancer cells [23]. To verify MLH1 is a direct target of *miR-148b*, we cloned the 3’-UTR of MLH1 containing the single putative *miR-148b*-binding site downstream of the Renilla luciferase open reading frame. Both wild-type 3’-UTR and a mutant form, in which the putative seed-binding site was mutated, were evaluated using luciferase assay (Figure 3A). As shown in Figure 3(B), co-transfection of *miR-148b* precursor with wild-type MLH1 3’-UTR reporter construct significantly repressed relative luciferase activity whereas mutation of the *miR-148b*-binding site eliminated this effect in A549 cells (Figure 3B). On the other hand, co-transfection of *miR-148b* inhibitor with wild-type MLH1 3’-UTR reporter construct into A549 cells significantly induced relative luciferase activity which was reversed when the *miR-148b*-binding site was mutated (Figure 3C). In addition, transfection of *miR-148b* mimic or inhibitor decreased and increased MLH1 protein level in A549 cells (Figure 3D). Taken together, these results demonstrate that *miR-148b* can directly regulate MLH1 expression level.

**Figure 3:** *miR-148b* directly targets the 3’-UTR of MLH1 and regulate its expression level in lung cancer cells (**A**) The wild-type 3’-UTR of mammalian MLH1 mRNA contains a putative *miR-148b*-binding site. The mutant form was shown below. (**B** and **C**) Luciferase reporter assays. A549 cells were transfected with reporters containing the wild-type or mutant form after transfection with control miRNA as well as *miR-148b* mimic or inhibitor respectively. Data represent the mean ± S.D. *, *P*<0.05; **, *P*<0.01. (**D**) Western Blot analysis of MLH1 protein level in A549 cells transfected with control, *miR-148b* mimic or inhibitor. β-Actin was used as loading control.

RETRACTED

### *miR-148b* mediates radiosensitivity through regulating MLH1 protein expression

To determine the importance of MLH1 in the regulatory role of *miR-148b* in radioresistance, we ectopically express MLH1 in A549 cells transfected with *miR-148b* mimic (Figure 4A). Although transfection of *miR-148b* mimic reversed radioresistance, overexpression of MLH1 eliminated this sensitizing effect (Figure 4B). Additionally, stable knockdown of MLH1 in A549 cells phenocopied the effect of *miR-148b* overexpression by sensitizing these cells to irradiation (Figures 4C and 4D). These results suggest that MLH1 is required for the regulatory role of *miR-148b* in radioresistance.

**Figure 4:** *miR-148b* mediates radiosensitivity through regulating MLH1 protein expression (**A**) Western Blot analysis of MLH1 protein level in A549 cells transfected with control or *miR-148b* mimic or *miR-148b* plus MLH1 cDNA. β-Actin was used as loading control. The MLH1 to β-actin ratio is 1:0.12:1.8. (**B**) Clonogenic survival in cells described in (A) after exposure to 2, 4 or 8 Gy of γ-radiation. Survival was normalized to unirradiated control cells. Student's *t* test was used to compare the difference between control and *miR-148b* mimic group. (**C**) Western Blot analysis of MLH1 protein level in A549 cells expressing control or MLH1 shRNA. β-Actin was used as loading control. The MLH1 to β-actin ratio is 1:0.23. (**D**) Clonogenic survival in cells described in (C) after exposure to 2, 4 or 8 Gy of γ-radiation. Survival was normalized to unirradiated control cells. (**B** and **D**), data represent mean ± S.D., *n*=3. *, *P*<0.05; **, *P*<0.01.

### Up-regulation of *miR-148b* decreases A549 cell radioresistance *in vivo*

To validate the regulatory role of *miR-148b* in radioresistance *in vivo*, we examined the effects of *miR-148b* inhibition on radioresistance of A549 cells using xenograft mouse model. As shown in Figures 5(A)–5(C), transfection with *miR-148b* mimic significantly reduced tumour size, inhibited tumour growth and reduced tumour weight. Immunohistochemistry (IHC) analysis showed that the *miR-148b* mimic transfected xenografts showed significantly increased cleaved caspase 3 compared with the control xenografts (Figure 5D). Taken together, these results suggest that *miR-148b* can regulate radioresistance *in vivo*.

**Figure 5:** Up-regulation of *miR-148b* decreases A549 cell radioresistance *in vivo* (**A**) Image of representative tumours from control or *miR-148b* mimic transfected A549 xenografts 3 weeks after exposure to 8 Gy of γ-radiation. (**B**) Tumour growth curve of control or *miR-148b* mimic injected A549-IR tumours. *n*=5 for each group. (**C**) Weights of tumours from mice described above at sacrifice. (**D**) Representative cleaved caspase 3 IHC staining of xenografts from the two groups in (C). The bar graph presents the quantification of IHC staining. The scale bar indicates 100 μm. Data represent mean ± S.D. **, *P*<0.01; ***, *P*<0.001.

RETRACTED

## DISCUSSION

Acquisition of resistance to radiotherapy represents a major obstacle in the treatment of NSCLC. It is known to significantly increase the morbidity and mortality of NSCLC patients. Therefore, identification of effective therapeutic strategies which can sensitize the NSCLC to radiotherapy is urgently needed to enhance survival rate in NSCLC. In the present study, we identified a panel of altered miRNAs in a radioresistant NSCLC cell line A549, after IR exposure and analysed the expression level of one of the top candidates, *miR-148b* in clinical human samples (Supplementary Figure S1). We observed that *miR-148b* was down-regulated in both serum and tissues from NSCLC patients compared with healthy controls. It is also down-regulated in radioresistant NSCLC patient samples compared with radiosensitive patient samples (Figure 1). These observations suggest that *miR-148b* may serve as a potential predictive biomarker for radiotherapy in NSCLC.

A growing body of evidence has suggested that there is a link between a collection of miRNAs and radioresistance and those miRNAs function as either radiosensitizers or radioprotectors through various mechanisms. For example, *miR-23* and *miR-203* have been shown to enhance radiosensitivity by targeting IL8/Stat3 and IL8/AKT signalling pathway, respectively in nasopharyngeal carcinoma [24,25]; *miR-205* has been reported to function as a tumour radiosensitizer by inhibiting DNA repair pathway via down-regulation of ZEB1 and Ubc13 in breast cancer cells [26]; *miR-15a/16* can enhance radiation sensitivity of NSCLC cells by targeting the TLR1/NF-κB signalling pathway [27]. On the other hand, it has been reported that *miR-106b* can induce cell radioresistance via the PTEN/phosphoinositide 3-kinase (PI3K)/AKT pathways and p21 in colorectal cancer [28]; *miR-20a* has been recently shown to induce cell radioresistance by activating the PTEN/PI3K/AKT signalling pathway in hepatocellular carcinoma.

Several reports have supported that *miR-148b* is down-regulated in many cancer types, including NSCLC and may function as a tumour suppressor [16–18]. Additionally, *miR-148b* has been shown to reverse cisplatin resistance in NSCLC and is up-regulated after IR exposure in human endothelial cells [20,21]. However, its role in regulating radioresistance has not been investigated. In the present study, we found that overexpression or inhibition of *miR-148b* could increase or decrease radiosensitivity in NSCLC cells by regulating DNA repair pathway (Figure 2). Importantly, expression of *miR-148b* mimic significantly inhibited tumour growth after IR exposure in A549 xenograft with resultant increased apoptotic cell death (Figure 5).

RETRACTED

Radiotherapy leads to the production of a variety of ionizing radiation-induced lesions in DNA, which are required to be repaired by DDR pathways, including DNA single-strand breaks (SSBs), DNA DSBs, DNA base alterations and DNA–DNA or DNA–protein cross-links [29]. Over the past decade, a variety of approaches have been employed to target DDR components for radiosensitization, including small interfering RNA, aptamers, antisense and small molecule inhibitors [30–33]. MLH1 is a protein involved in mismatch repair (MMR) pathway and genetic or epigenetic modification in this gene results in microsatellite instability (MSI) [34]. Accumulating evidence suggests that DNA MMR proteins may influence and/or are directly involved in the DDR following radiation induced DSBs and MSI cancers with deficiency in those proteins may indicate sensitivity to radiotherapy [35]. Our results showed that *miR-148b* can directly bind to the 3’-UTR of MLH1 and manipulation of *miR-148b* expression affected MLH1 protein level (Figure 3). Additionally, knockdown of MLH1 sensitized A549 cells to irradiation, phenocopying the effect of *miR-148b* down-regulation (Figure 4A). Overexpression of MLH1 reversed the radiosensitizing effects of *miR-148b* mimic (Figure 4B). These results suggest that *miR-148b* exerts its radiosensitizing effects primarily through regulating MLH1 expression.

In the present study, we found that *miR-148b* was down-regulated in human NSCLC and radioresistant patient samples. Up-regulation of *miR-148b* sensitized radioresistant NSCLC A549 cells to IR by interfering DDR through down-regulating MLH1 protein level. These observations provide a rationale for the development of new therapeutic strategies to improve radiotherapy efficacy in lung cancer patients. *miR-148b* may represent a novel biomarker for the prediction of radiosensitivity in NSCLC.

## Abbreviations

DDR: DNA damage repair
DNMT1: DNA (cytosine-5)-methyltransferase 1
DSB: double-strand break
IHC: immunohistochemistry
MLH1: MutL homologue 1
MMR: mismatch repair
MSI: microsatellite instability
NSCLC: non-small cell lung cancer
